The article "MiR-520f promotes cell aggressiveness by regulating fibroblast growth factor 16 in hepatocellular carcinoma" was retracted in 2025. Reasons: plagiarized images; duplicated images; overlap with other authors' work.

# MiR-520f promotes cell aggressiveness by regulating fibroblast growth factor 16 in hepatocellular carcinoma

**DOI:** 10.18632/oncotarget.22726

**Published:** 2017-11-30

**Authors:** Feng Feng Xu, Wen Feng Xie, Guo Qing Zha, Hong Wu Chen, Liang Deng

**Affiliations:** ^1^ Department II of General Surgery, The Fifth Affiliated Hospital of Guangzhou Medical University, Guangzhou 510700, China; ^2^ Department of Intensive Care Unit, The Eastern Hospital of the First Affiliated Hospital, Sun Yat-sen University, Guangzhou 510700, China; ^3^ Upper Limb Department Of Orthopedics, The Eastern Hospital of the First Affiliated Hospital, Sun Yat-sen University, Guangzhou 510700, China; ^4^ Department of Emergency, The Eastern Hospital of the First Affiliated Hospital, Sun Yat-sen University, Guangzhou 510700, China; ^5^ Department of Hepatobiliary Surgery, The Seventh Affiliated Hospital, Sun Yat-sen University, Shenzhen 518107, China

**Keywords:** miR-520f, HCC, metastasis, FGF16

## Abstract

Cancer metastasis is a multistep cellular process, which has be confirmed one of mainly causes of cancer associated-death in hepatocellular carcinoma (HCC). MicroRNAs (miRNAs) participate in tumorigenesis function as either tumor suppressor genes or oncogenes. In order to elaborate the critical miRNAs and their targets in HCC, we compared the differential expression of miRNA between HCC tissues and normal tissues. Microarray analysis revealed there were several significantly up-expression miRNAs in HCC, compared to normal solid tissue. Among them, the expression of miR-520f was the most over-expression in HCC cell lines than that in human normal liver cells LO2, as well as up-regulated in HCC than that in the corresponding normal tissues. Moreover, Kaplan Meier-plotter analyses revealed that higher miR-520f levels were negatively correlated with poor overall survival. By applying bioinformatics methods to identify the targeting genes of miRNA, we demonstrated that fibroblast growth factor 16 (FGF16) was the miR-520f-targeted gene. Meanwhile, FGF16 exhibited similar expression patterns to miR-520f in HCC. Forced miR-520f expression accelerated HCC cells proliferation and aggressiveness *in vitro* and *in vivo*, whereas down-regulation of miR-520f caused an opposite outcome. Moreover, over-expression of FGF16 was closely related to the metastatic potential of HCC cells. Herein, we also confirmed that ectopic expression of FGF16 in HCC cells promoted proliferation, colony formation, and increased migration, invasion of HCC cells *in vitro*. Collectively, our results indicated that over-expression of miR-520f and FGF16 was positively associated with aggressive phenotypes and poor survival of patients with HCC, and miR-520f promoted HCC aggressive phenotypes by regulating the expression of FGF16. MiR-520f may be employed as a prognostic factor and therapeutic target for HCC.

## INTRODUCTION

As one of the most lethality and aggressive cancer, hepatocellular carcinoma (HCC) has been proven is the major cause of cancer mortality in worldwide [1]. The stage of HCC at diagnosis is an efficient prognostic factor of clinical outcomes, but, there approximately 20∼30% of HCC patients are possess un-resectable distant diffusion [2]. Overall survival (OS) of HCC patients closely dependents on the occurrence of locally aggressive and distant metastasis [3]. Hence, better investigations of the molecular mechanisms in relation to HCC metastasis can bring about potential prognostic marker and target for the combat of HCC metastasis [4].

MiRNAs, which are 18-22 non-coding RNAs, regulate proteins expression by post-transcriptionally and extensive molecular mechanisms in various cancer types via either oncogenic or tumor-suppressive activities [5]. Substantive reports have indicated that the levles of miRNAs during the progression of colorectal cancer (CRC) altered, which highlighted their crucial roles for disease diagnostic and prognostic of CRC [6]. On account of the comprehensive roles of miRNAs in tumor genes regulation and cellular processes, investigation of miRNAs that accelerate tumor aggressiveness and predict of cancer prognosis is of interest.

Growth factors are the crucial stimulators of tumor occurrence and development upon binding to receptors that expressed on tumor cell surface. Fibroblast growth factor (FGF), which is identified in fibroblasts, constitutes a family of growth factors in various multi-cellular organisms [7]. Apart from wound healing and normal tissues development, FGFs are implicated in multitudinous cellular functions, including cells apoptosis, cells survival, differentiation and mobility [8]. Furthermore, substantial evidences validate that FGF signaling pathway is association with the progression of malignant cancers. Fibroblast growth factor 16 (FGF16), which is a 207-amino acid protein, contains a vital region of 120 amino acids that binds to FGF receptor (FGFR3) and heparin [9]. Although originally characterized in the rat, FGF16 has been demonstrated that be expressed preferentially in brown adipose tissue and participated in the proliferation of brown adipocytes in zebrafish [10]. Furthermore, in the embryonic mouse, previous research reveal the vital function of FGF16 in cardiac myocyte proliferation and development of coronary vasculature [11]. Nevertheless, the association of FGF16 with HCC growth and metastasis has not been well elaboration.

In this current study, we reported that miR-520f was remarkably up-regulated in HCC cells and clinical tissues, and was associated with the clinical prognosis of HCC. Overexpression of miR-520f promoted the growth and metastasis of HCC cells. Our findings imply that miR-520f plays pivotal oncogenic roles in HCC progression and hints its potential as a therapeutic target for HCC.

## RESULTS

### miR-520f is up-regulated in HCC

To investigate the difference pattern of miRNAs in HCC, we analyzed the miRNA expression profiles in normal tissues compared to HCC [12]. 32 miRNA genes were remarkably over-expressed in HCC compared to normal tissues (Figure 1A and Supplementary Table 1). The microarray meta-analysis (http://ngs.ym.edu.tw/ym500v2/) revealed miR-520f is the most significantly up-expressed in HCC compared with normal. The similar findings were also found in clinical HCC tissues. The level of miR-520f was remarkably increased in 58 cases of HCC samples, as compared to normal tissues by qRT-PCR (Figure 1B). Next, we explored the clinical outcomes of HCC patients with different level of miR-520f. Of relevance, we found that patients possess high level of miR-520f exhibited a poor overall survival (Figures 1C and Supplementary Table 2). Finally, the similar results were also obtained in the four HCC cell lines, among which miR-520f level is higher in HCC cell lines than LO2 cells (Figure 1D). All results suggested that miR-520f was positively associated with malignancy of HCC.

**Figure 1:** The expression of miR-520f in HCC cell lines and HCC tissues **(A)**. YM500v2 microRNA meta-analysis (http://ngs.ym.edu.tw/ym500v2/index.php) was used to compare miRNA in HCC and non-cancerous tissues. The hierarchical clustering of differentially expressed miRNAs among HCC and normal tissues was shown. Group 1: Normal, Group 2: HCC. **(B)**. The level of miR-520f was detected by qRT-PCR in 58 cases of HCC tissues and 27 corresponding normal tissues. **(C)**. Survival analysis was conducted to assess the prognostic value of miR-520f in overall survival (OS) of patients with HCC. **(D)**. qRT-PCR analysis was applied to determine the level of miR-520f in four HCC cell lines. PCR values of genes were normalized to UBC. Data were presented as the mean ± SD. For indicated comparisons, ^**^ *P* < 0.01.

### FGF16 is a target of miR-520f

To investigate the mechanisms responsible of miR-520f for HCC growth and metastasis, bioinformatics analyses were performed to search for miR-520f targets. Three target genes prediction websites (Targetscan, PicTar and miRDB) were applied to predict the potential targets of miR-520f. Notably, 11 genes (TNFAIP1, FGF16, CXXC5, TMEM74, RASSF2, ZNF2, PPAP2B, MYCBP, LETMD1, UBXN1 and ACTBL2) were present in the all databases (Figure 2A). Among these candidate genes, we focused on FGF16 owing to it has been demonstrated to be involved in tumorigenesis of several cancer types [13]. To further verify that miR-520f directly target 3′UTR of FGF16 gene, the interaction between the 3’UTR of FGF16 and miR-520f was validated by luciferase analysis. The luciferase activities in the reporter containing the 3′-UTR of WT FGF16 was significantly suppressed, whereas miR-520f mimic had no obviously inhibition effect on the luciferase activities of reporter containing 3′-UTR of MUT FGF16 (Figure 2B and Supplementary Figure 1). Next, we verified whether the expression of FGF16 was regulated by miR-520f in HepG2 and PLC/PEF/5 cells. As shown in Figure 2C and 2D, the levels of FGF16 were assessed in HepG2 and PLC/PEF/5 cells that were transfected with miR-520f mimic or miR-520f inhibitor. Overexpression of miR-520f decreased the mRNA level of endogenous FGF16 in both HepG2 and PLC/PRF/5 cells. Conversely, inhibition of miR-520f significantly increased FGF16 levels in HepG2 and PLC/PRF/5 cells. Conditioned medium collected from HCC cells transfected with miR-520f mimic or mimic-NC was subjected to ELISA. As shown in Figure 2E, the secreted FGF16 in medium were reduced in miR-520f over-expressing HepG2 and PLC/PEF/5 cells. Immunofluorescence assays future demonstrated that FGF16 was markedly inhibited in HepG2 cells that transfected with miR-520f, and was elevated in HepG2 upon transfected with miR-520f inhibitor (Figure 2F and 2G). In addition, analysis the level of miR-520f and FGF16 in HCC tissues exhibited a positively correlation (Figure 2H) and these results were consistent with HCC cell lines. Meanwhile, both qRT-PCR and immunoblotting assays showed FGF16 was remarkably over-expression in HCC cells, as compared with LO2 cells (Figure 2I). Immunohistochemical staining demonstrated that FGF16 was notably over-expressed in HCC tissues, when compared to corresponding normal tissues (Figure 2J). Finally, we found that HCC patients with high level of FGF16 possessed a shorter overall survival (Figure 2K). Taken together, all these results strongly suggest that FGF16 is a target of miR-520f in HCC.

**Figure 2:** FGF16 is directly modulated by miR-520f **(A)**. Schematic presentation of miR-520f target prediction by silico analyses. Venn diagrams indicated candidate genes determined by three prediction algorithms. **(B)**. The wide-type (WT) and mutant (MUT) 3′-UTR region of FGF16 were fused with luciferase reporter and co-transfected with miR-520f mimic or NC mimic into 293T cells. The luciferase assay revealed that miR-520f bind to the 3′-UTR region of WT FGF16. Each bar represents the relative luciferase activity. **(C)**. The mRNA level of FGF16 was remarkably increased when HepG2 and PLC/PRF/5 cells transfected with miR-520f mimic.^**^ *P* < 0.01 compared to NC-mimic. **(D)**. The mRNA level of FGF16 in both HCC cells was significantly decreased after cells were transfected with miR-520f inhibitor. ^**^ *P* < 0.01 compared to NC inhibitor. **(E)**. ELISA analysis of the secreted FGF16 levels in medium after HCC cells transfected with miR-520f mimic. ^**^ *P* < 0.01 compared to NC-mimic. **(F)**. The levels of FGF16 were significantly increased after HepG2 cells transfected with miR-520f mimic as shown in immunofluorescence assay. Scale bar represents 200 μm. **(G)**. FGF16 in HepG2 cells were inhibited after cells transfected with miR-520f inhibitor. Scale bar represents 50 μm. **(H)**. The expression of miR-520f was positively related to the level of FGF16. **(I)**. The levels of FGF16 in HCC cell lines were markedly increased as compared to LO2 cells as assayed by qRT-PCR (left panel) and immunoblotting analysis (right panel). ^**^ *P* < 0.01 compared to LO2 cells. **(J)**. Compare to normal tissues, the significantly higher FGF16 level was observed in HCC tissues. Scale bar represents 200 μm. **(K)**. Survival analysis evaluated the prognostic value of FGF16 in OS of patients with HCC.

### MiR-520f impairs aggressiveness of HepG2 and PLC/PRF/5 cells

To uncover the potential roles of miRNA-mediated growth, migration and invasion in HCC cells, HepG2 and PLC/PRF/5 were transfected with miR-520f or miR-520f inhibitor. Intriguingly, cell proliferation assays suggested that HepG2 and PLC/PRF/5 cells upon transfected with miRNA mimic exhibited higher proliferative capacity and colony formation than the control cells (Figure 3A and 3B). The HepG2 and PLC/PRF/5 cells transfected with miR-520f inhibitor showed lower growth and clone formation, as compared to control (Figure 3C and 3D). In the wound-healing assay, the wound closure was smaller in miR-520f-transfected HCC cells than that in control cells after 24 h (Figure 3E). In contrast to miR-520f over-expression, we found larger width in healing of miR-520f inhibitor transfected HCC cells (Figure 3G). In Transwell analysis, miR-520f obviously accelerated the invasive of HCC cells (Figure 3F). As expected, inhibition effects on invasion were discovered in miR-520f inhibitor transfected HCC cells (Figure 3H). These findings indicated miR-520f played a role in HCC cell growth, mobility and invasion *in vitro*.

**Figure 3:** Effect of miR-26 on the aggressiveness of HepG2 and PLC/PRF/5 cells **(A)**. CCK-8 cells proliferation assay. **(B)**. Colony formation analysis revealed transfection of miR-520f mimic in HepG2 and PLC/PRF/5 cells accelerate cellular progression. ^**^ *P* < 0.01 compared to NC-mimic. **(C)**. CCK-8 assay. **(D)**. Colony assay revealed transfection of miR-520f inhibitor in HepG2 and PLC/PRF/5 cells reduce cellular growth *in vitro*. ^**^ *P* < 0.01 compared to NC-mimic. **(E)**. Wound closure assay revealed that miR-520f mimic increased the cellular mobility of HepG2 and PLC/PRF/5 *in vitro*. Scale bar represents 500 μm. ^**^ *P* < 0.01 compared to NC-mimic. **(F)**. Transwell assay shown that miR-520f over-expression increased the invasion of HepG2 and PLC/PRF/5 *in vitro*. Data were presented as the mean ± SD from three independent measurements. Scale bar represents 50 μm. ^**^ *P* < 0.01 compared to NC-mimic. **(G)**. Wound-healing assay was performed to determine the effect of miR-520f inhibitor in HepG2 and PLC/PRF/5 cellular mobility *in vitro*. Scale bar represents 500 μm. ^**^ *P* < 0.01 compared to NC-mimic. **(H)**. Transwell assay suggested that transfection of miR-520f inhibitor in HepG2 and PLC/PRF/5 inhibited cells invasion *in vitro*. Data were presented as the mean ± SD. Scale bar: 50 μm. ^**^ *P* < 0.01 compared to NC-mimic.

### MiR-520f impairs aggressiveness of HCC cells dependent on FGF16

To explore whether FGF16 reversed the roles of miR-520f in HCC cell aggressiveness, we manipulated the expression of FGF16 in HepG2 and PLC/PRF/5 cells that ectopic expression of miR-520f. We found that down-expression of FGF16 effectively inhibited clone formation and metastasis in HCC cells that transfection with miR-520f (Figure 4A-4C). On the other hand, ectopically expression of FGF16 resulted in a markedly FGF16 levels increase in HCC cells that pre-transfection with miR-520f inhibitor. As expected, up-regulation of FGF16 rescued miR-520f inhibitor-mediated growth and metastasis in HepG2 and PLC/PRF/5 cells (Figure 4D-4F). Altogether, these findings indicated that FGF16 was a **core element** which mediated miR-520f-induced pro-tumor effects in HCC.

**Figure 4:** FGF16 reverses the effect of miR-520f-mediated HCC cell aggressiveness **(A)**. Down-regulation of FGF16 in miR-520f mimic transfected HCC cells inhibited colonies formation. **(B)**. Wound healing revealed down-expression of FGF16 markedly decreased cells migration upon transfection with miR-520f mimic. Scale bar represents 500 μm. **(C)**. Transwell invasion revealed down-expression of FGF16 markedly decreased cells invasion upon transfection with miR-520f mimic. Scale bar represents 500 μm. Data were presented as the mean ± SD. ^**^ *P* < 0.01 compared to control. ^##^ *P* < 0.01 compared to miR-520f + shCTL. **(D)**. The effect of miR-520f inhibitor on colony formation was reversed by over-expression of FGF16 in HepG2 and PLC/PRF/5 cells. Values shown were mean ± SD. **(E)**. Wound healing revealed over-expression of FGF16 significantly increased cells migration upon transfection with miR-520f inhibitor. Scale bar represents 500 μm. **(F)**. Transwell invasion revealed over-expression of FGF16 significantly increased cells invasionupon transfection with miR-520f inhibitor. Scale bar represents 500 μm. Data were presented as the mean ± SD. ^**^ *P* < 0.01 compared to control.^##^ *P* < 0.01 compared to miR-520f + vector.

### FGF16 regulates aggressiveness of HepG2 and PLC/PRF/5 cells

Because miR-520f regulated the protein expression of FGF16, we next investigated whether FGF16 exert a direct regulation on the aggressiveness of HCC. As shown in Figure 5A, both HepG2 and PLC/PRF/5 cells that subjected to FGF16 knocked-down, exhibited down-expression of FGF16 compared to the controls. The down-regulation of FGF16 restrained HepG2 and PLC/PRF/5 proliferation, colony formation and migration, invasion and tube formation of human umbilical vein endothelial cells (HUVECs) (Figure 5B-5E). Furthermore, FGF16 down-expression exerted a negative effect on the tumor growth of HepG2 and PLC/PRF/5 cells *in vivo* (Figure 5F). Immunohistochemical staining suggested the expressions of FGF16 and Ki67 were suppressed in the tumor tissues that formed by FGF16 down-regulation HCC cells (Figure 5G). In addition, HepG2 and PLC/PRF/5 cells that transfected with vector containing FGF16 exhibited higher expression of FGF16 compared to control cells (Figure 6A). As expected, FGF16 over-expressing HepG2 and PLC/PRF/5 cells possessed more remarkably proliferation, metastasis and promoted tube formation of HUVECs (Figure 6B-5E). Finally, subcutaneously inoculation of FGF16 over-expressing cells accelerated the tumorigenic potential of HepG2 and PLC/PRF/5 cells *in vivo* (Figure 6F). Consistently, immunohistochemical revealed higher expression of FGF16 as well as Ki67 in tumor mass derived from FGF16 over-expressing cells compared with those in tumors formed by control cells (Figure 6G). Taken together, all these results suggested that FGF16 regulated the growth and aggressiveness of HCC cells.

**Figure 5:** Effect of FGF16 on invasiveness and tumorigenesis of HCC cells **(A)**. The levels of FGF16 were decreased in HepG2 and PLC/PRF/5 cells by FGF16 shRNA transfection. **(B)**. The cell proliferation was compared in HepG2 and PLC/PRF/5 shFGF16 and HepG2 and PLC/PRF/5 control cells based on CCK-8 assay (left panel) and colony formation (right panel). **(C)**. The ability of migration was compared in HepG2 and PLC/PRF/5 shFGF16 and indicated control cells based on wound healing assay. Scale bar represents 500 μm. **(D)**. The ability of invasion *in vitro* was compared in HepG2 and PLC/PRF/5 shFGF16 and control cells based on Transwell invasion assay. Scale bar represents 50 μm. **(E)**. Tube formation assay of was conducted to compare the tube formation of HUVECs that treated with HepG2 and PLC/PRF/5 shFGF16 culture medium (CM) or control cells medium. Scale bar represents 200 μm. **(F)**. A decrease of mean tumor volume in mice group with HepG2 and PLC/PRF/5 shFGF16 tumors was observed, as compared to the control group. **(G)**. Reduced regulation of Ki67 was also shown by immunohistochemical staining in xenograft tumors derived from HepG2 and PLC/PRF/5 shFGF16 cells. Scale bar represents 200 μm. Data are presented as the mean ± SD from three independent measurements. ^**^ *P* < 0.01 compared to shCTL.

**Figure 6:** Effect of FGF16 over-expression on HCC cell invasiveness and tumorigenesis **(A)**. The levels of FGF16 were increased in both HepG2 and PLC/PRF/5 cells after transfected with FGF16. **(B)**. The proliferation was compared in FGF16 over-expressing HCC cells and control cells based on CCK-8 assay (left panel) and colony formation (right panel). **(C)**. The ability of migration was compared in FGF16 over-expressing HepG2 and PLC/PRF/5 and control cells based on wound healing assay. Scale bar represents 500 μm. **(D)**. The ability of invasion *in vitro* was compared in FGF16 over-expressing HepG2 and PLC/PRF/5 and their control cells based on Transwell invasion assay. Scale bar represents 50 μm. **(E)**. Tube formation assay was applied to determine the tube formation of HUVECs that treated with HepG2 and PLC/PRF/5 FGF16 over-expressing culture medium (CM) or control cells medium. Scale bar represents 200 μm. **(F)**. An increase of mean tumor volume in mice group with ectopic expression of FGF16 in HepG2 and PLC/PRF/5 tumors was observed, as compared to the control group. **(G)**. Up-regulation of Ki67 was also shown by immunohistochemical staining in xenograft tumors derived from HepG2 and PLC/PRF/5 FGF16 over-expression cells. Scale bar represents 200 μm. Data were presented as the mean ± SD. ^**^ *P* < 0.01 compared to vector.

### MiR-520f impairs aggressiveness of HCC cells in *in vivo*

Lastly, we examined the roles of miR-520f in HCC cells growth and dissemination *in vivo* by using nude mice models of HCC. Firstly, miR-520f over-expressing HCC cells were implanted subcutaneously into nude mice. Remarkably, miR-520f over-expressing HCC cells formed solid tumor mass in the inoculation site (Figure 7A). Immunohistochemical staining showed higher level of Ki67 in miR-520f over-expressing tumor tissues compared to the control tumor tissues (Figure 7B). Subsequently, we utilized the xenograft model wherein the miR-520f over-expression HCC cells were injected via tail-vein. As expected, the mice injected with miR-520f over-expressing cells possessed a greater degree of metastasis loci (Figure 7C). The biological effects of miR-520f down-expression on HCC progression were also further examined using a xenograft tumor model. As showed in Figure 7D, tumors formed by miR-520f down-expressing cells exhibited a smaller size and mass than tumors formed by the control cells. Immunohistochemical staining assays suggested the regulatory role of miR-520f down-expressing on proliferation index Ki67 in the tumor tissues (Figure 7E). To future determine whether miR-520f down-expression resulted in the inhibition of HCC cells metastasis *in vivo*, the parental or miR-520f inhibitor transfected HCC cells were injected into mice via vein tail, and metastasis loci was determined five weeks later. Histologic analysis revealed the number of metastatic lesions formed by miR-520f inhibitor cells was significantly reduced (Figure 7F). Taken together, these findings indicated that miR-520f contributed to HCC cells growth and metastatic *in vivo*.

**Figure 7:** The effect of miR-520f on malignant progression of HCC cells *in vivo* **(A)**. Tumor growth kinetics (mean ± SD) of cells that transfected with miR-520f mimic versus control cells in nude mice. **(B)**. Ki67 was detected in xenograft tumors. Data were presented as the mean ± SD. ^**^ *P* < 0.01, compared to NC-mimic. Scale bar, 200 μm. **(C)**. Representative images of H&E-stained lung from mice injected with control cells or miR-520f over-expression cells. Scale bar, 200 μm. ^**^ *P* < 0.01, compared to NC-mimic. **(D)**. HepG2 and PLC/PRF/5 cells transfected with miR-520f inhibitor or control cells were implanted in nude mice. Tumor volumes were measured on the indicated days. **(E)**. Ki67 was detected by immunohistochemical staining in xenograft tumors. Data were presented as the mean ± SD. ^**^ *P* < 0.01, compared to NC inhibitor. Scale bar, 200 μm. **(F)**. Representative images of H&E-stained lung from mice injected with control cells or cells transfected with miR-520f inhibitor. Data were presented as the mean ± SD. Scale bar, 200 μm. ^**^ *P* < 0.01, compared to NC inhibitor.

## DISCUSSION

MiRNAs have been demonstrated play a crucial part in tumorigenesis and metastasis of hepatocellular carcinoma (HCC) [14]. Illustration the underlying molecular mechanisms of miRNA in HCC may improve therapeutic strategies for HCC patients. In this study, we identified the over-expression of miR-520f in clinical HCC tissues and HCC cell lines. Furthermore, miR-520f regulated HCC growth and metastasis partly via regulating FGF16, and altered the expression of FGF16 reversed the effect of miR-520f in HCC growth and metastasis.

Cumulative evidence suggests dys-regulated miRNAs participate in oncogenesis, cellular metastasis and survival of HCC [15]. Our research revealed differential expression of miRNAs in HCC and the microarray data shown 37 miRNAs (32 up-regulations and 7 down-regulations) that were differentially expressed between human HCC and normal tissues. Several dys-regulated miRNAs which identified in this study are associated with cancer progression [16], suggesting common underlying molecular mechanisms during cancer cells metastasis. Herein, we identified miR-520f to be up-regulated in HCC cell lines and HCC tissues in our data.

MiRNAs have emerged as critical regulators of the occurrence and development of malignant tumor by targeting multiple cancer-associated genes. Although miR-520f has not been linked to EMT or invasion before, it has been described to play a vital role in drug resistance [17, 18]. In human pancreatic cancer PANC-1 cells, miR-520f enhanced sensitivity to gemcitabine. Furthermore, miR-520f increased the sensitivity of a cisplatin resistant neuroblastoma cell line to etoposide and cisplatin [19]. Nevertheless, the clinical significance of alter miR-520f and the molecular mechanisms of miR-520f underlying the HCC metastasis remains not well investigations. Down-expression of miR-520f in HCC cell resulted in the inhibitory effects growth and metastasis both *in vitro* and *in vivo*. In contrast, ectopic expression of miR-520f promoted the growth and metastasis ability of HCC cells. Three target genes prediction websites were performed to predict target genes and we found that FGF16 was one of the direct targets of miR-520f. Previously, FGF16 has been demonstrated to be over-expressed in breast carcinoma and its expression positively correlates with metastasis through regulating multiple transcription factors and up-regulating the expression of integrin alpha-5, colony stimulating factor 1 (CSF-1), stromal cell-derived factor 1 (SDF-1) and C-X-C motif chemokine receptor 4 (CXCR4) [10]. Furthermore, FGF16 promotes angiogenesis in breast cancer by simultaneously enhancing hypoxia-inducible transcription factor 1α (HIF1α) and activator protein-1 (AP-1) mediated vascular endothelial growth factor A (VEGF-A) transcription [20]. Besides, FGF16 expression was identified to have prognostic significance in head and neck carcinoma. However, the role and clinical significance of FGF16 in HCC has not been well investigated.

In the current study, forced expression of FGF16 pheno-copied the effects of miR-520f over-expression in HCC cells, which sustaining a role of miR-520f in regulating FGF16 expression in HCC. Moreover, we found the positive relationship between miR-520f and FGF16 expression in HCC, which corroborated the biological relevance of miR-520f/FGF16 network in HCC. Subsequently, we demonstrated that FGF16 over-expression strikingly restored cell growth, mobility and invasion phenotypes in HCC cells that pre-transfected with miR-520f inhibitor. Knocked-down of FGF16 reversed the effects of miR-520f over-expression in HCC cell proliferation and aggressiveness. In conclusion, our research identifies the potential mechanism underlying the pro-tumor growth and metastasis of miR-520f/FGF16 axis in HCC.

## MATERIALS AND METHODS

### Cell culture and clinical samples

HCC cell lines (HepG2, SNU-423, SNU-387, SNU-449, Bel-7402 and PLC/PRF/5) were obtained from the Chinese Academy of Sciences Cell Bank of Type Culture Collection (CBTCCCAS, Shanghai, China). HCC cell lines were cultured in DMEM or 1640 medium supplemented with 10% FBS, 100 μg/ml streptomycin and 100 U/ml penicillin, maintained at 37 °C with CO_2_. Normal liver cells LO2 used as control were obtained from CHI Scientific (Jiangyin Jiangsu, China) and was cultured in DMEM medium supplemented with 20%fetal bovine serum, 100 μg/ml streptomycin and 100 U/ml penicillin, maintained at 37 °C with CO_2_. Human umbilical vein endothelial cells (HUVECs) were obtained from CHI Scientific (Jiangyin Jiangsu, China) and were cultured in 1640 medium supplemented with 20%fetal bovine serum. The study and informed consent were certified by the Ethics Committee of the Fifth Affiliated Hospital of Guangzhou Medical University. The informed consents were acquired from each enrolled patient. 58 patients (31 males and 27 females) with HCC, who received no chemotherapy or radiation treatment prior to surgery, were enrolled from November 2008 to July 2016. 58 cases of cancer tissues and 27 cases of normal tissues were collected after patients received surgical removal and preserved in liquid nitrogen.

### Meta-analysis of miRNA expression in HCC

The online database YM500v2 (http://ngs.ym.edu.tw/ym500v2/) was applied to analyze the differential miRNA in HCC and normal tissues. The YM500v2 compared the miRNA pattern between 50 cases of normal tissues and 147 cases of HCC tissues, and a total of 2578 miRNAs were analyzed. In total, 37 miRNAs were significantly changed in the HCC compared to the normal (32 were up-regulated, and 5 were down-regulated). Among the 32 up-regulated, 3 miRNAs were determined to be up-regulated by an infinite fold change at an extremely low expression level in the normal group and miR-520f ranked first among them.

### Cell transfection

Short hairpin RNA (shRNA) targeting FGF16 (shFGF16), scrambled shRNA (shCTL), miR-520f/normal control (NC) mimic, and miR-520f/NC inhibitor were synthesized by GenePharma (Shanghai, China). HepG2 and PLC/PRF/5 cells were transfected with miR-520f mimic, miR-520f inhibitor or shFGF16 utilized Lipofectamine^®^ 2000 Transfection Reagent (Invitrogen). Full-length human FGF16 complementary DNA (cDNA) was amplified by PCR and cloned into pcDNA3.1 (+) expression vector (Invitrogen) and then transfected into cells using Lipofectamine^®^ 2000 Transfection Reagent (Invitrogen) according to the manufacturer’s instructions [21].

### CCK-8 proliferation assay

Cell proliferation was performed using cell counting kit-8 (CCK-8) (KeyGEN, Nanjing, China). Firstly, cells (1 × 10^3^/well) were seeded into 96-well plates and cultured for 24, 48 and 72 h. Then, 10 μl CCK-8 solutions were added into each well. After 2 h, the absorbance (450 nm) was determined using a microplate reader [22].

### Colony formation assay

1 × 10^3^ single-cell suspension was plated into 6-well plates. Cells were cultured in medium containing 10% FBS, with 2 ml fresh medium changed every three days for total 21 days. The cells colonies were stained with 0.1% crystal violet and counted.

### Wound healing analysis

The migration ability of cells was assessed using the wound closure assay. 3 × 10^5^ cells/well was plated into 6-well plates. After 24 h, cells formed monolayer confluence. A scratch was created with a 100-μl pipette tip. Cell debris was removed with phosphate-buffered saline (PBS) and cultures were supplemented with medium for 24 h. Migration images were captured by an inverted microscope (Carl Zeiss, Oberkochen, Germany) and the relative percentage of wound closure was determined by comparing to control cells [23].

### Tanswell invasion assay

Invasion analysis was conducted by Transwell inserts with polycarbonate membranes (8.0 μm pore size) with Matrixgel (BD). 4 × 10^4^ cells were seeded into the upper chamber and culture medium containing 20% FBS was added in the lower chamber. After 6 h, the invaded HCC cells on the lower surface of the membrane were stained with 0.1% crystal violet and counted in 5 random fields [24].

### Tube formation assay

24-well plates were pre-coated with Matrigel (BD). 4 × 10^3^ cells/well human umbilical vein endothelial cells (HUVECs) were seeded into wells and were incubated with culture medium from indicated HCC cells. Three days later, the total tube length formed by HUVECs per image field was analyzed.

### Luciferase assay

3′-UTR of wild-type (WT) FGF16 and mutant (MUT) FGF16 were specifically synthesized (Promega) and inserted into the pmirGLO dual-luciferase miRNA target expression vector. 5 × 10^4^ cells/well 293 T cells were seeded into 24-well plates. The miR-520f mimic with pmirGLO-FGF16 3′-UTR WT vector or pmirGLO-FGF16 3′-UTR MUT vector were co-transfected into 293T cells using Lipofectamine^®^ 2000. After 48 h, luciferase assays were assessed by using the dual luciferase reporter assay system (Promega) [25].

### Enzyme-linked immunosorbent assay (ELISA)

The levels of FGF16 in conditioned medium were detected by ELISA kits (AMEKO, LianShuo biological, shanghai, China). Conditioned medium was diluted with the sample dilution buffer with a ratio of 1:1. Standard curves were created using purified FGF16 and the CurveExpert 1.3 software program.

### Western blot analysis

Equal total protein were separated on SDS-PAGE and transferred onto PVDF membrane. The membrane was blocked with 5% non-fat dry milk and then incubated with anti-FGF16 antibody (Santa Cruz Biotech) or anti-GAPDH antibody (Santa Cruz Biotech). Then, membrane was incubated with HRP-conjugated secondary antibody (Santa Cruz Biotech) and protein bands were detected using ECL western blotting kit (Amersham Biosciences, UK) [26].

### Quantitative real-time PCR

Total RNA was isolated from HCC cells or HCC samples using the RNeasy Mini Kit (QIAGEN, USA), and cDNA was synthesized using QuantiTect Reverse Transcription Kit (QIAGEN, USA). The level of miR-520f was assessed through mirVanaTM qRT-PCR microRNA Detection Kit (GeneCopoeia) and the mRNA of FGF16 was determined using SYBR Green quantitative Real-time PCR Master Mix kit in Biosystems 7300 Real-Time PCR system (ABI, Foster City, CA, USA). Relative quantities of miR-520f and FGF16 were calculated using 2^(-ΔΔCt)^ method. The primers used for PCR were as follows (sense and antisense, respectively): FGF16: 5’-GTACAACACCTATGCCTCAACC-3’ and 5’-TCTTTGTTCAGGGCCACGTAA-3’; UBC: 5’-GGGGCACCTCCTATGAGAGAT-3’ and 5’-TCCCTCCGCAGTTTCTTCCA-3’; miR-520f: 5’-ACACTCCAGCTGGG CCTCTAAAGGGAAGCG-3’ and 5’-CTCAACTGGTGTCGTGGAGTCGGCAATTCAGTTGAGAGAAAGCG-3’

### Immunofluorescence

HCC cells grown on glass coverslips for 24 h and were fixed with 3.7% formaldehyde, and permeabilized with 0.1% Triton X-100. Then, the coverslips were incubated with antibody against FGF16 (Santa Cruz Biotech) for 24 h at 4 °C. After 24 h, the coverslip was washed with PBS for twice and was incubated with the secondary FITC antibody. Finally, the coverslip was incubated with 4, 6-diamino-2-phenylindole (DAPI) for staining the nuclear.

### *In vivo* tumorigenicity assay

100 μl 1 × 10^6^ cells were inoculated subcutaneously into the flank of 5-week-old female athymic nude mice (n=6 for each group). Tumor size was monitored each three days by detecting the length (L) and width (W). Tumor size was calculated according to the formula: (length × width^2^)/2. All nude mice were killed under anesthesia after inoculation 25 days [27].

### Tail vein metastasis model

1.5 × 10^6^ cells were re-suspended in PBS and were injected into athymic nude mice via tail vein. Mice were sacrificed 5 weeks after injection for cells. Lung tissues were collected and subjected to histology staining and examination [28].

### Immunohistochemical staining assays

The xenograft tumor tissues were fixed in 4% paraformaldehyde and embedded in paraffin. 3 μm paraffin section were incubated with FGF16 or Ki67 antibodies (Santa Cruz Biotech) at 4 °C overnight. The secondary streptavidin-HRP-conjugated antibody staining (Santa Cruz Biotech) was performed at room temperature for 1 h. Finally, the paraffin sections was counterstained with hematoxylin [29].

### Statistical analysis

Each assay was conducted in three independent experiments. Data were expressed as means± standard deviation (SD). Student’s t-test was applied to evaluate the results of two groups. *P* < 0.05 was considered as statistically significant.

## SUPPLEMENTARY MATERIALS FIGURE AND TABLES


